# Reprogramming glioblastoma multiforme cells into neurons by protein kinase inhibitors

This article has been retracted.

**DOI:** 10.1186/s13046-018-0857-5

**Published:** 2018-08-02

**Authors:** Jie Yuan, Fan Zhang, Dennis Hallahan, Zhen Zhang, Liming He, Ling-Gang Wu, Meng You, Qin Yang

**Affiliations:** 1 Cancer Biology Division, Department of Radiation Oncology, Washington University School of Medicine, 4511 Forest Park, St. Louis, MO 63108 USA; 2 Medical Center of Stomatology, the First Affiliated Hospital of Jinan University, Guangzhou, 510630 China; 3 School of Stomatology, Jinan University, Guangzhou, 510630 China; 4 Synaptic Transmission Section, National Institute of Neurological Disorders and Stroke, Bethesda, MD 20892 USA

**Keywords:** GBM, mTOR, Neuron, Protein kinase inhibitors, Reprogramming, ROCK

## Abstract

**Background:**

Reprogramming of cancers into normal-like tissues is an innovative strategy for cancer treatment. Recent reports demonstrate that defined factors can reprogram cancer cells into pluripotent stem cells. Glioblastoma multiforme (GBM) is the most common and aggressive malignant brain tumor in humans. Despite multimodal therapy, the outcome for patients with GBM is still poor. Therefore, developing novel therapeutic strategy is a critical requirement.

**Methods:**

We have developed a novel reprogramming method that uses a conceptually unique strategy for GBM treatment. We screened a kinase inhibitor library to find which candidate inhibitors under reprogramming condition can reprogram GBM cells into neurons. The induced neurons are identified whether functional and loss of tumorigenicity.

**Results:**

We have found that mTOR and ROCK kinase inhibitors are sufficient to reprogram GBM cells into neural-like cells and “normal” neurons. The induced neurons expressed neuron-specific proteins, generated action potentials and neurotransmitter receptor-mediated currents. Genome-wide transcriptional analysis showed that the induced neurons had a profile different from GBM cells and were similar to that of control neurons induced by established methods. In vitro and in vivo tumorigenesis assays showed that induced neurons lost their proliferation ability and tumorigenicity. Moreover, reprogramming treatment with ROCK-mTOR inhibitors prevented GBM local recurrence in mice.

**Conclusion:**

This study indicates that ROCK and mTOR inhibitors-based reprogramming treatment prevents GBM local recurrence. Currently ROCK-mTOR inhibitors are used as anti-tumor drugs in patients, so this reprogramming strategy has significant potential to move rapidly toward clinical trials.

**Electronic supplementary material:**

The online version of this article (10.1186/s13046-018-0857-5) contains supplementary material, which is available to authorized users.

## Background

The ability to convert somatic cells into disease-relevant cell types through cellular reprogramming has opened new doors for basic research and cell replacement therapy [1]. Takahashi et al. demonstrated that defined factors could drive skin-derived fibroblasts to induced pluripotent stem (iPS) cells that could be further differentiated into the desired cell type. Direct somatic lineage reprogramming has attracted much attention as it bypasses conversion into iPS cells. Recently studies have demonstrated that a set of neural factors can directly convert fibroblasts into neurons [2–11]. Direct fibroblast-neuron reprogramming provides an alternative, potentially complementary tool to many of the proposed applications of iPS technology for both disease modeling and development of cell-based therapies.

Reprogramming healthy somatic cells with defined factors has been extensively investigated. However, reprogramming cancer cells has comparatively lagged behind [12–14]. Differentiation of tumors into post-mitotic cells is an ancient idea. For example, tretinoin (all-trans-retinoic acid) was used as differentiation therapy of acute promyelocytic leukemia [15]. Recent established reprogramming method should significantly improve differentiation therapy. Reprogramming and oncogenic transformation are stepwise processes that share many similarities. Overexpression of a set of oncogenes induces reprogramming and oncogenic transformation, while tumor suppressor gene such as p53 suppresses both processes. Although unidentified biological barriers may exist [14, 16, 17], reprogramming of both solid and liquid tumors to iPS cells has been reported by different groups [16, 18–27]. Loss of tumorigenicity by unknown mechanisms and induced dedifferentiation to pluriopotency seem to be common features of reprogrammed cells from different cancers. However, robust differentiation into specific lineages remains a stumbling block [28–32]. To overcome these roadblocks, therefore, we will detect whether cancer cells can be reprogrammed into normal-like cells under defined reprogramming conditions.

Glioblastoma multiforme (GBM) is the most common and most aggressive malignant primary brain tumor in humans. Despite multimodal therapy [surgery with ionizing radiation and chemotherapy (temozolomide, TMZ)], the outcome for patients with GBM is still poor, with a median survival of only 14 months [33–35]. Therefore, it is imperative to develop novel therapeutic strategies for GBM treatment. Integration-free reprogramming of cancer cells is a safe and preferable strategy for clinical use. We screened a kinase inhibitor library and found that a combination of two inhibitors, Rho-associated protein kinase (ROCK) and mammalian target of rapamycin (mTOR), could substitute for transcription factors and convert human GBM cells into neural-like cells. The induced neural cells were subsequently trans-differentiated into functional neurons. The induced neurons lost their tumorigenicity and reverted to the ‘normal state’. Importantly, ROCK-mTOR inhibitors coupled with reprogramming treatment prevented GBM local recurrence in mice, suggesting that our reprogramming treatment had a key role in preventing GBM recurrence.

## Methods

### Cell culture

Human GBM cells, U118, GM97 and PDC1 were routinely cultured in 60 mm dish (MidSci) in Dulbecco’s modified Eagle medium (Hyclone) containing 10% fetal bovine serum (Millipore-Sigma), non-essential amino acids (Invitrogen) and penicillin/streptomycin (Invitrogen) at 37 °C in 5% CO_2_. U118 and GM97 have *p53* mutation or inactivation (p53 data base, p53.fr), while U118 also carries *pten* mutation [36]. Human fibroblasts IMR90 from ATCC are lung-derived fibroblasts from a 16-week fetus. All cell lines have been tested for mycoplasma infection and were authenticated by short tandem repeat DNA profiling analysis.

### Neural cell conversion

For neuronal conversion, GBM cells were plated at a density of 3.0 × 10^4^ cells cm^− 2^ on microscope glass coverslips coated with matrigel (BD) in 35 mm dishes. For neural induction, the media was changed to defined induction medium including DMEM/F12 (2% FBS) plus 1 μM dexamethasone (Millipore-Sigma), 0.5 mM isobutylmethylxanthine (Millipore-Sigma), 200 μM indomethacin (Millipore-Sigma), 2 μM Y-27632 (Enzo Life Sciences) and 2 μM P529 (Millipore-Sigma). For kinase inhibitor screening experiments, we used 2 μM protein kinase inhibitor from a library (Calbiochem, 355 inhibitors). For neuronal differentiation, we used neuronal mature medium including Neural medium (ScienCell) with 50 μM dbcAMP (Millipore-Sigma), 10 ng/ml NT3 (PROSPEC), 10 ng/ml BDNF (PROSPEC), 0.5 μM Retinoic acid (Millipore-sigma), 2 μM Y-27632 and 2 μM P529. Quantitative of mean % induced neuron (iN) purity is counted by morphology of MAP2-positive staining, and numbers represent the percentage of iN cells at the time point of quantification.

### Cortical neuron culture and co-culture with iNs

Primary cortical neurons were isolated from P0 rats. Cortices were dissected and dissociated by trypsin digestion (0.25% Trypsin, 137 mM NaCl, 5 mM KCl, 7 mM Na_2_HPO_4_, 25 mM HEPES) and plated on poly-D-lysine coated glass coverslips. The neurons were maintained in growth medium consisting of MEM supplemented with B27, glutamine (all from Invitrogen), glucose, transferrin (Calbiochem), fetal bovine serum and Ara-C (both from Millipore-Sigma) for a week before co-culture with iNs. iNs were induced for 7 days by induction medium with P + Y and dissociated by trypsin (0.05% Trypsin). iNs were seeded onto a cortical neuron bed and maintained in neuronal mature medium.

### Viral preparation, western blot and immunofluorescence

ROCK1/2 and mTORC1 (Raptor) /C2 (Rictor) shRNAs were obtained from Millipore-Sigma. Western blotting analyses were performed to check the knockdown efficiency. Immunofluorescence staining was performed as follows: 5 × 10^4^ modified human fibroblasts were planted on Matrigel-coated glass coverslips the day before induction. Cells were fixed for 20 min at room temperature in 4% paraformaldehyde in PBS, permeabilized for 30 min in PBS containing 0.2% Triton X-100 and 10% normal goat serum (NGS) and incubated overnight at 4 °C in PBS containing 10% NGS and primary antibodies. Cells were washed three times with PBS and incubated for 2 h at room temperature with anti-rabbit or anti-mouse secondary antibodies conjugated to Alexa Fluor-488 or Alexa Fluor-594 (1:500, Invitrogen). Images were acquired on immunofluorescence microscope or Zeiss LSM 510 META confocal microscope at 40× magnification and 1.3 numerical aperture oil-immersion objective.

The following antibodies were used for the immunofluorescence studies: rabbit anti-MAP2 (Millipore-Sigma, 1:200), mouse anti-Tuj1 (R&D Systems, 1:100), rabbit anti-synapsin 1 (Cell Signaling, 1:200), mouse anti-TUJ1 (1:1000, Covance) and rabbit anti-Tuj1 (1:2000, Covance).

### Trypan blue dye exclusion assays, qRT-PCR and TUNEL assays

GBM, iP and iN cells were seeded at a density of 10,000 cells/well in a 12-well plate. Cells were counted with a ViCell cell viability analyzer (Beckman Coulter). Cell proliferation was normalized to the percentage of control cells. Three independent experiments were performed with triplicates for each cell line. For qRT-PCR assay, total RNA was extracted using Trizol isolation system (Invitrogen) according to the manufacturer’s instructions. Total RNA was treated with DNase I (Qiagen) to prevent DNA contamination. 2 μg RNA was reverse transcribed using Transcriptor High Fidelity cDNA Synthesis Kit (Roche). Reverse transcription and real-time PCR were performed as a standard procedure. The terminal deoxynucleotidyltransferase-mediated dUTP-biotin nick end labelling (TUNEL) assay was performed with TUNEL assay kit (Roche).

### Electrophysiology

Coverslips plated with iNs were placed in the recording chamber mounted on an Olympus 1 × 81 microscope. All electrophysiology recordings were recorded at room temperature (22–25 °C) via whole-cell recording with a patch electrode. Signals were amplified using Heka EPC-10 amplifier and filtered at 2 KHz via a Bessel low-pass filter. Data were sampled using Puls8.8 software, and analysed using Igor6.04.

For recording voltage-gated currents and action potentials, patch electrodes were filled with solution (in mM): 130 K-gluconate, 10 KCl, 10 HEPES, 0.5 EGTA, 4 MgATP, 0.3 Na2GTP, 10 P-Creatin, pH adjusted by KOH to 7.2, osmolarity measured at 310 mOsm. The composition of the external solution used for recording was as follows (in mM): 105 NaCl, 25 NaHCO3, 3 Myo-Inositol, 2 Na-Pyruvate, 2.5 KCl, 1.25 NaH2PO4, 25 Glucose, 2 CaCl2, 1.5 MgCl2, pH adjusted by NaOH to 7.4, osmolarity measured at 300 mOsm. To isolate voltage-dependent sodium currents, 1 μM tetrodotoxin was added to the external solution. To monitor voltage-gated currents, we applied step potentials ranging from − 60 mV to + 60 mV for 20 ms. To monitor action potentials, we applied step currents ranging from 10 to 100 pA for 200 ms. External solution changes were achieved rapidly, within 100 ms.

### Microarray analysis

Microarray analysis was performed at the Washington University Genome Center. Briefly, Illumina HumanHT-12 v4 Expression BeadChip was used and samples were labeled by biotin. The Direct Hybridization Assay was performed and the data were scanned on the BeadArray Reader. Scanned images were quantitated by Illumina Beadscan, v3. Quantitative data was imported into Illumina GenomeStudio software and normalized by Illumina’s quantile method. The quantile-normalized background-subtracted data were calculated in excel. Data were filtered based on the average signal with baseline set as 50. Only the genes with division value > 3 were selected and considered as differentially expressed. All differentially expressed genes were clustered using MeV software.

Gene expression for each sample was analyzed to determine the relationship among GBM cells and iNs. Data were filtered based on average signal and baseline was set as 10 to increase the sensitivity. Differentially expressed genes were identified with a 3-fold change as the threshold. To examine the potential neuron differentiation pathways relevant to immortalization, all neuron differentiation genes from Gene Ontology Website (http://www.geneontology.org/, GO: 0030182) were compared with the microarray data. For gene enrichment analysis, we used web-based Gorilla program (http://cbl-gorilla.cs.technion.ac.il/). Thus, these results will greatly help for understanding mechanisms of GBM cell reprogramming.

### GBM and iN cell transplantation and GBM recurrence treatment in mice

We implanted GBM cells and iNs in the corpus callosum of nude mice. On the day of transplantation, cells were harvested with accutase, counted, and re-suspended at concentration of 25,000 cells/μL. Four microliter cell suspension was injected into the corpus callosum of mice using the following stereotactic co-ordinates (in reference to Bregma point): 10.98 mm (anterio-posterior axis), 21.75 mm (latero-medial axis) and 22.25 mm (vertical axis). Control GBM cells were injected into left side and iNs were injected into right side of the same mouse. Mice with cell transplants were perfusion fixated at 2 weeks, 1 month and 4 months. Brains were excised and sectioned on a cryostat for IHC analysis of the cell implants. The primary antibodies used are described above. Subsequently, various secondary antibodies were used to visualize the specific primary immunoreaction product in single and double IHC staining. For GBM local recurrence experiments, we used a mouse model of local recurrence following surgical resection of orthotopic GBM tumors [37–40]. GBM tumors generated by GM97 cells in nude mice were surgically removed after 4 weeks when the primary tumors had reached ~ 50 mm^3^. 95% of each tumor was excised and a small fragment of tumor, the largest being 2 mm^3^, was not removed to model postoperative residual GBM. Matrix-Driven Delivery (MDD) Pellet of ROCK-mTOR inhibitors with dried induction medium was prepared by Innovative Research of America. We implanted the MDD pellet including mTOR-ROCK inhibitors (2 μM P + Y, 5 μl per day for 21 days) with or without dried induction medium into the resection cavity of GBMs. MDD pellet with dried induction medium, pellet only and no treatment were controls. Induction media in each MDD pellet include 1 μM dexamethasone, 0.5 mM isobutylmethylxanthine and 200 μM indomethacin with 105 μl DMEM/F12 (2% FBS). Mouse brains were excised and sectioned on a cryostat for IHC and TUNEL assay analyses.

## Results

### Screening a protein kinase inhibitor library to reprogram GBM cells

Reprogramming somatic cells are into iPS cells by transcription factors may cause genomic instability, which increases the risk of cancer-cell induction [41–45]. Therefore, we tried to develop a transgene-free method to efficiently reprogram GBM cells into normal-like cells. Cellular senescence has been shown to regulate reprogramming fibroblasts to iPS cells and fibroblast-neuron conversion [46–49]. Since many protein kinases are involved in senescence and proliferation processes, we screened a protein kinase inhibitor library (355 inhibitors, Calbiochem). We prepared a GBM cell line (U118) with expression of MAP2 promoter-RFP. Through phenotypic change screening, we found that candidate kinase inhibitors reprogrammed GBM cells into induced progenitor-like cells in induction medium (Fig. 1a, b). We observed that a subpopulation of cells was MAP2-RFP positive with marked morphological changes after 3–7 days in induction medium with candidate kinase inhibitor treatment. Cell morphology ranged from large nuclear and flat shaped cells (cancer cells) to small, bipolar cells, termed induced neural-like cells (Fig. 1a,b). Eight candidate small molecules/compounds were selected for further confirmation (Fig. 1c). Secondary screening confirmed that three compounds induced morphological changes with higher efficiency (Fig. 1c). Two candidate small molecules, namely rapamycin and palomid 529 (P529), are mTOR inhibitors and the third one (Y27632) is a ROCK inhibitor. To determine the combinatorial effects of these inhibitors on GBM-neural cell conversion, we found that using mTOR-ROCK inhibitors (P529/Y27632) together converted GBM cells into neural-like cells with the highest efficiency (~ 90% induced efficacy after 7 days induction) (Fig. 1c).

**Fig. 1:** Protein kinase inhibitor screen for reprogramming GBM cells. **a** & **b** Screening design and primary screening results. Human GBM cells (U118) expressing MAP2-promoter-RFP were seeded in 96-well plates. Kinase inhibitors were added at a final concentration of 2 μM in the induction medium. The medium was changed every other day until day 7 when cells converted to RFP-positive cells. Images were taken on day 7 after inhibitor treatment. Positive induced neural-like cells were counted by RFP-positive staining and quantified on day 7. The histogram represents the ratio of normalized data for kinase inhibitor treatment as compared with DMSO. **c** Secondary screening results. U118 cells were treated with candidate kinase inhibitors. R + Y: Rapamycin+Y27632; P + Y: P529 + Y27632. Quantitative data are the mean ± SEM from three independent experiments

To investigate whether ROCK-mTOR inhibitors have a general effect on human GBM cells, another GBM cell line (GM97) and one patient-derived primary GBM cell (PDC1) were treated with ROCK-mTOR inhibitors. After induction for 3–7 days, about 70–90% of these GBM cells converted into neural-like cells (Additional file 1: Figure S1). Thus, reprogramming treatment of ROCK-mTOR inhibitors is able to convert multiple GBM cells into neural-like cells.

### Reprogramming GBM cells into induced neurons

Next, we examined whether the GBM cells could be reprogrammed into another lineage (neuron, a lineage switch) in a defined neuronal medium. After 3 days in neuronal medium with mTOR-ROCK inhibitors, induced neural-like cells further differentiated into bi- or multi-polar neuron-like cells. In 2–3 weeks, 70–90% of GBM U118 cells converted to neurons with mature neuronal morphology that expressed the neuronal markers, Tuj1 and MAP2 (Fig. 2a & c). We calculated the iN yield as the percentage of MAP2+ cells in relation to the initial number of plated GBM cells. At 3 weeks after induction, we obtained yields of 90 ± 15% (Fig. 2a). In contrast, after 4 weeks in neuronal medium without kinase inhibitors, control GBM cells maintained GBM cell morphology with negative staining of MAP2 (Fig. 2b). Furthermore, we verify the neuron induction in two other GMB cells, GM97 and PDC1. Three weeks after induction, ~ 75–90% of GBM cells converted into iNs (Additional file 1: Figures. S1-S2). Moreover, iNs did not express astrocyte (GFAP) and oligodendrocyte marker (O4) (Additional file 1: Figure S3). These results suggest that ROCK-mTOR inhibitor treatment led to conversion of GBM cells to neurons.

**Fig. 2:** ROCK-mTOR inhibitors induce GBM-Neuron cell conversion. **a** Kinetic analysis of iNs from GBM U118 cells was performed after induction with ROCK-mTOR inhibitors in neuronal medium. The bar graph shows quantity of iN cells with MAP2 positive staining. Quantitative data are presented as mean ± SEM from three independent experiments. **b** No expression of MAP2 and Synapsin in U118 control cells without reprogramming treatment. **c** Expression of TUJ1, MAP2, Synapsin, LHX6 and TBR1 was examined in iNs 3 weeks after induction. B & C: Nuclei were counterstained with DAPI (blue). Scale bar, 10 μm. **d-f** Electrophysiological characterization of U118 cells was performed 3 weeks after induction. **d** Representative traces of membrane currents were recorded with a ramp protocol (lower panel, a voltage ramp from -80 mV to + 60 mV over 500 ms). Fast activating Na + currents were prominent. **e** Representative current traces (upper panel) were recorded in voltage-clamp mode. Cells were depolarized by voltage steps from − 60 to + 60 mV in 10-mV increments (Δ10mV, upper panel). The lower panel shows the current-voltage (I-V) relationship for sodium current. **f** Sample traces of spontaneous synaptic currents (without pharmacological blockers) were recorded at a holding potential of − 80 mV

So far, we identified iNs based on their morphology and positive staining of several neuronal markers. Next, we further characterized the functional aspects of iNs induced by ROCK-mTOR inhibitor treatment from GBM U118 cells. We found that ~ 80% of iNs showed Synapsin-positive puncta that label the vesicles in the presynaptic nerve terminal (Fig. 2c). Furthermore, iNs showed positive immunostainings with TBR1 (60%) or LHX6 (55%), indicating that iNs have properties of different neuronal populations present in the forebrain (Fig. 2c).

To determine whether iNs generate action potentials and neurotransmitter-induced currents, the basic functions of neurons, we cultured U118 cells (7 days post-induction) with a monolayer culture of primary rat neurons, which might provide a better environment for maturation [2, 3]. Three weeks after co-culture, whole-cell voltage-clamp recordings of iNs showed that 70% of iNs exhibited inward fast activating and inactivating sodium currents and outward potassium currents during a ramp depolarization. This was also confirmed by applying a series of voltage steps to evoke inward sodium currents and outward potassium currents (Fig. 2d, e, 70% positive efficacy, *n* = 30). Miniature excitatory postsynaptic currents were recorded from induced neurons without co-culture, suggesting that iNs can form functional synapses by themselves (Fig. 2f, 65% positive efficacy, *n* = 30). These data indicate that iNs are functional neurons.

We also tested the effects of reprogramming treatment on normal primary neurons and astrocytes. We prepared primary mouse neurons/astrocytes and found that the reprogramming treatment of mTOR-ROCK inhibitors did not affect neuron/astrocyte properties under drug concentration for reprogramming (Additional file 1: Figure S4). These data indicate that normal neurons/astrocytes are only marginally responsive to our treatment strategy.

### Genome-wide transcriptional profiling of induced neurons

To analyze the similarities between iNs and parental GBM cells, we performed microarray-based comparative global gene expression profiling. Microarray data was quantile normalized and filtered based on the average signal, and differently expressed genes were selected for further analysis. Hierarchical cluster analysis revealed a significant difference between iN cells and their parental GBM U118 cells (Fig. 3a, b). The clustering analysis of global gene expression revealed that iNs from GBM cells by the reprogramming treatment of ROCK-mTOR inhibitors are particularly similar to control neurons, which are induced from fibroblasts by p53 knockdown (Fig. 3b) [49]. This indicates that iNs generated by different methods show similarity of gene expression profiling. Using the Ontology Data-base for enrichment analysis, we found that the key factors involved in neuron differentiation were significantly changed in iNs, compared with those in parental GBM cells. Moreover, we examined mRNA levels of key factors reported to be involved in neuron conversion. We found that, in iNs induced by the reprogramming treatment of ROCK-mTOR inhibitors, expressions of a set of neurogenic transcription factors were increased by > 10-fold (Fig. 3c), suggesting that these factors may be involved in GBM-neuron conversion. These findings indicate that genetic trans-differentiation erases majority of the expression hallmarks of the cell of origin, while specifically inducing the neuronal phenotype.

**Fig. 3:** Global gene expression profiling of GBM and iNs. **a** Heat-map of differentially genes expressed was generated for GBM U118 (WT) and iNs. Positive control neurons are induced from IMR90 fibroblasts by p53 knockdown [49]. **b** Hierarchical clustering was performed. **c** qRT-PCR results show relative mRNA levels of defined transcription factors in GBM U118 control and iNs (*n* = 3)

### ROCK1/2 and mTORC1 shRNAs generate iNs

Both ROCK and mTOR are serine/threonine protein kinases. ROCK is a kinase belonging to the AGC (PKA/PKG/PKC) family, including ROCK1 and ROCK2 [50–53]. mTOR interacts with other proteins and serves as a core component of two protein complexes, mTOR complex 1 and mTOR complex 2 [54–60]. To determine if ROCK and mTOR pathways are involved in GBM-neuron conversion, we examined the effects of ROCK and mTOR knockdown on GBM-neuron conversion (Fig. 4a). Lentiviral constructs expressing short hairpin RNA (shRNA) against ROCK1/2 and mTORC1 (Raptor)/C2 (Rictor) were transfected into GBM U118 cells. We found that knockdown of ROCK1, ROCK2 or mTORC1 (Raptor) could reprogram GBM cells into neural-like cells, while knockdown of mTORC2 did not (Fig. 4b). Combination treatment of ROCK1/2 and mTORC1 shRNAs converted GBM cells to neural-like cells with kinetics and conversion efficiency similar to ROCK-mTOR inhibitors. Moreover, the iNs showed typical neuronal morphology and positive immunostaining for neuronal markers TUJ1, MAP2 and Synapsin. Efficiency of neuronal conversion by shRNA treatment was similar to ROCK-mTOR inhibitors (Fig. 4c & d). Thus, we conclude that ROCK1/2 and mTORC1 kinases are involved in conversion of GBM to neurons.

**Fig. 4:** Effects of ROCK1/2 and mTORC1 shRNAs on GBM cell conversion. **a** Western blot analysis from U118 cells showed that shRNA1 and shRNA2 of ROCK1/2 and mTORC1 (Raptor) /C2 (Rictor) are sufficient to inhibit ROCK1/2, Raptor or Rictor expression, respectively. Expressions of downstream targets pS6 for Raptor and pAKT1-S473 for Rictor were reduced by Raptor or Rictor shRNAs. R1: ROCK1, R2: ROCK2. **b** GBM U118 cells were transduced with ROCK1/2 and mTOR1/2 shRNAs and then cultured in induction medium. Positive induce neural cells were counted using RFP-positive staining and quantified on day 7. The histogram represents the ratio of normalized data between treatment with shRNAs or DMSO. R1: ROCK1, R2: ROCK2, m1: mTORC1. **c** Kinetic analysis was performed for iNs after induction with ROCK1/2-mTORC1 shRNAs in induction medium (induction for the first week) and neuronal mature medium (induction after 1 week). iN cells was quantified as MAP2 positive cells. Quantitative data are the mean ± SEM from three independent experiments. **d** Expression of TUJ1, MAP2 and Synapsin in iNs was examined 3 weeks after induction with ROCK1/2-mTORC1 shRNAs. Scale bar, 10 μm

### Loss of proliferation and tumorigenicity in iNs

We performed proliferation assays to determine iN cell proliferation. Trypan blue exclusion assays were performed after treating cells with ROCK-mTOR inhibitors. We observed that ROCK-mTOR inhibitor treatment reduced cell proliferation in time-dependent manner in GBM cells, but not in iNs (Fig. 5a and Additional file 1: Figures S5A & S6A). In addition, apoptosis increased in GBM cells upon ROCK-mTOR inhibitor treatment, but not in iNs (Fig. 5b and Additional file 1: Figures S5B & S6B). These data suggest that ROCK-mTOR inhibitor treatment does not affect iN cell proliferation and survival, but may mediate GBM cell proliferation by regulating apoptosis.

**Fig. 5:** Proliferation and invasion ability of iNs. **a** GBM GM97 and iN (3 weeks induction) cells were treated with 2 μM P + Y. Proliferating cells (viable) were evaluated by trypan blue dye exclusion assay at day 4 after treatment. Shown are the mean fold change in cell number relative to the 24-h time point and SEM from three treatments. **b** TUNEL assay was performed for GBM GM97 and iN cells treated with 2 μM P + Y. Apoptotic cells were evaluated at day 4 after treatment from three treatments. Etoposide treatment (5 μM) was used as a positive control. **c-e** GBM GM97 and iN cells were seeded for soft agar assays (**c** & **d**) and invasion assays (**e**). Quantitative data are the mean ± SEM from three independent experiments

We further evaluated cell proliferation and invasion. The mature phenotype of iNs was accompanied by cessation of proliferation and invasion as measured by soft-agar proliferation and invasion assays (Figs. 5c-e and Additional file 1: Figure S6C & S6D). To determine tumorigenic properties in vivo, we injected parental GBM cells and iNs (1.5 × 10^5^) into the brain frontal lobe, 2 mm lateral to the bregma of nude mice (Fig. 6a) [49]. No tumors were formed following iN transplantation up to 16 weeks (Fig. 6b). Transplantation of GBM cells treated with induction medium without ROCK-mTOR inhibitors resulted in tumor formation in 10 of 10 mice after 4 weeks. Thus, we conclude that reprograming GBM cells to neurons can abrogate the parental tumor cell tumorigenicity.

**Fig. 6:** Reprogramming orthotopic GBMs in mice. **a** Experimental design for tumor formation in mice. **b** Parental GBM cells (Control) and iNs were implanted into the same nude mice (left and right side each mouse, respectively) and the tumor formation was measured. **c** & **d** GBM tumors generated by GM97 cells in nude mice with postoperative recurrence model. ROCK-mTOR inhibitors (P529 and Y27632, P + Y) with induction media in the MDD pellet were administered directly into the resection cavity of GBMs. P + Y without induction medium, medium only (both in the MDD pellets) or no treatment were used as controls. Tumor recurrence (**c**) and mouse survival (**d**) were measured (*n* = 10). **e** Postoperative residual GFP-GBM were treated with ROCK-mTOR inhibitors (P + Y) with induction medium. GFP-positive cells expressed the mature neuronal markers MAP2 and Synapsin 2 weeks after transplantation. Data are presented as mean ± SEM from 5 mice (300 cells/section and 2 sections per mouse were counted). The scale bar represents 10 μm. **f-g** Ki67 (IHC) and apoptotic (TUNEL assay) cells were evaluated in postoperative brain tissues treated with P + Y and induction media. Normal brain tissue was as the control. Ki67 and apoptotic cells from recurred tumors treated with P + Y without induction media, media only or no treatment were also examined. Scale bar 10 μm

### Reprogramming orthotopic intracranial GBM prevents local recurrence

Despite advances in varieties of treatment modalities for GBM, local relapse remains a clinically significant problem. We examined whether our reprogramming treatment could prevent GBM local recurrence using a mouse model [37–40]. GBM tumors were generated by transplanting GFP-GM97 cells in nude mice. After four weeks, when primary tumors had reached ~ 50 mm^3^, ~ 95% of each tumor was excised except for a small fragment (2 mm^3^). This fragment was not removed to model residual tumor cells after surgery. Matrix-Driven Delivery (MDD) Pellet of ROCK-mTOR inhibitors with dried induction medium was prepared by Innovative Research of America. The finished pellet had a biodegradable matrix that effectively and continuously releases the active product in the animal for three weeks. We implanted the mTOR-ROCK inhibitors with or without induction medium in the MDD pellet into the resection cavity of xenografts. Controls included no treatment, induction medium only and ROCK-mTOR inhibitors without induction medium in the MDD pellet. Tumor recurrence and mouse survival were measured (Fig. 6c, d, *n* = 10). Tumor recurrence was not observed up to 12 weeks in mice treated with mTOR-ROCK inhibitors with induction medium treatment (0/10 mice, Fig. 6c). Local recurrence was observed within 3–4 weeks in 10 of 10 mice without treatment or with induction medium only (Fig. 6c). 8/10 mice displayed tumor recurrence in mTOR-ROCK inhibitors without induction medium, suggesting that there is only a weak effect on GBM when using mTOR-ROCK inhibitors alone (direct chemotherapy). Immunohistochemistry (IHC) analysis revealed that 90% ± 5 of GFP/MAPs2 and 70% ± 8 of GFP/synapsin positive cells were detected 2 weeks after mTOR-ROCK inhibitor treatment with induction medium (Fig. 6e). These results suggest that GFP-GBM cells converted into mature neurons in vivo. Recurred tumors were examined from mTOR-ROCK inhibitors without induction medium, medium only or no treatment. It was observed that GFP-positive cells did not express MAP2 (Additional file 1: Figure S7). Tumors from mTOR-ROCK inhibitor treatment without induction medium had fewer Ki67 positive cells and more apoptotic cells as compared with tumors from medium only or no treatment control (Fig. 6f-g). Taken together, these results indicate that that mTOR-ROCK inhibitors under the reprogramming condition play a key role in preventing GBM local recurrence.

## Discussion

Collectively, we screened a kinase inhibitor library and found that a combination of the ROCK-mTOR kinase inhibitors can substitute for all transcription factors to reprogram GBM cells. This conversion is highly efficient, fast, and yields mature neurons. Induced neurons lose their tumorigenicity and reprogramming treatment prevents GBM local recurrence in mice. Reprogramming GBM by kinase inhibitors is a transgene-free method and ROCK-mTOR inhibitors have been used in patients. We believe that our findings will assist in the development of GBM therapy.

ROCK1 and ROCK2 have tissue-specific expression patterns. ROCK1 is mainly expressed in lung, liver, spleen, kidney and testis, while ROCK2 is distributed mostly in brain and heart. By acting on the cytoskeleton, ROCK regulates cell shape and movement, cellular immortalization and differentiation [50–53]. mTOR regulates cell growth, proliferation, protein synthesis, and transcription [54–60]. ROCK inhibitors are already used as anti-tumor drugs in patients, while mTOR inhibitors are used to prevent transplant rejection, promote longevity, and treat cancer in clinical trials. Thus, of ROCK-mTOR inhibitors-based reprogramming strategy is expected to have low risk in vivo and may rapidly move towards clinical trials. GBM cell lines used in this study also have *p53* mutation or inactivation*.* In future studies, we will examine the effects of *p53* on GBM reprogramming. Among the various proteins involved in the mTOR pathway, much interest in GBM has coated SGK1 kinase. Recently, a new SGK1 kinase inhibitor has shown good antiproliferative, proapoptotic capacity and synergistic potential with radiotherapy in GBM in vitro and in vivo. [61, 62] It is interesting to determine whether SGK1 regulates GBM reprogramming.

One key issue with reprogramming therapy is that reprogrammed cells may be reverted back to GBM cells and form a tumor in vivo. We found that induced neurons do not show signs of further proliferation following 4 weeks in replacement of differentiation media with maintenance media. Although we did not observe that the reprogrammed cells revert back, we could not rule out reversal of reprogrammed cells into tumors. Additional experiments with genetically different samples and long-term in vivo observation are needed to address this issue. It is known that GBM cell lines are highly passaged cells that may not recapitulate the properties of primary GBM. We reprogrammed patient-derived primary GBM cells in vitro and in vivo. In the future studies, we will work on designing reprogramming strategies for patient-derived primary GBMs with different genetic background.

Delineating the molecular mechanism behind neural conversion will aid further development of the method. Gene expression analysis suggests that ROCK-mTOR may act as the “master regulator” to coordinate a set of defined factors in blocking cell reprogramming in physiological conditions. Consistent with this view, ROCK-mTOR controls both iPS reprogramming and neural conversion, implicating a general mechanism of reprogramming, where loss of ROCK-mTOR may generate lineage progenitors that develop complete and functional lineages in various induction media. In previous studies, we found that cellular senescence is a key step in the conversion of human fibroblasts into functional neural cells, including three neural lineages (astrocytes, neurons, and oligodendrocytes) [48, 49]. By genetically manipulating the senescence process, we have provided a new method for converting most human fibroblasts into neural cells in only 1–2 weeks. Both ROCK and mTOR are involved in senescence and proliferation processes, implicating that the reprogramming process may also be regulated through the kinase-senescence signaling pathways. We found that expressions of a set of neurogenic transcription factors, such as Neurod2, Ascl1 and Myt1l, were increased during GBM-neuron cell conversion. Neurod2 is significantly downregulated in GBM patients, which is involved in the p53 pathway [63]. Ascl1 and Myt1l suppress GBM tumorigenicity and are required for glioblastoma stem cells to undergo neuronal lineage differentiation [64–66]. Correlations of reprogramming factors and GBM tumorigenesis need further investigation using patient tissues.

The reprogramming-based therapy presents new avenues for the development of GBM therapeutics. ROCK-mTOR inhibitors are already used as anti-tumor drugs in patients with few or no side effects. We expect that neurons generated by ROCK-mTOR inhibitors are “safe” in vivo. However, it is been shown that aberrant synapse formation between implanted neurons of the wrong subtype and endogenous cells can lead to significant motor side effects in human clinical trials for Parkinson’s disease. We will identify the subtypes of our induced neurons and evaluate their functional properties in vivo. Our results also show that the reprogramming treatment with kinase inhibitors does not affect normal neurons and astrocytes, supporting the safety of our reprogramming strategy. We believe that our strategy is a novel, low risk, and effective method that can be combined with conventional therapy for clinical use.

## Conclusions

In this study, we have developed a novel cell reprogramming-based method for GBM treatment. We screened a kinase inhibitor library, and found mTOR and ROCK inhibitors are sufficient to reprogram GBM cells into “normal” neurons. In vitro and in vivo tumorigenesis assays showed that induced neurons lose tumorigenicity and this reprogramming treatment prevented GBM local recurrence in mice. The role of the ROCK-mTOR pathways in GBM reprogramming is entirely novel. ROCK-mTOR inhibitors are already used as anti-tumor drugs in patients and promise few or no side effects in reprogramming. Therefore, the reprogramming-based therapy will provide new avenues for development of therapeutics for GBM in patients.

## Additional file

Additional file 1: **Figure S1.** ROCK-mTOR kinase inhibitors reprogram GBM cells into iNs. **Figure S2.** ROCK-mTOR kinase inhibitors reprogram GBM cells into iNs. **Figure S3.** iNs did not express astrocyte and oligodendrocyte markers. **Figure S4.** Effects of mTOR-ROCK inhibitor treatment on normal primary neurons/astrocytes. **Figure S5.** iNs lose abilities of proliferation. **Figure S6.** Proliferation and invasion ability of iNs. **Figure S7.** Recurred tumors did not express MAP2. (DOC 6831 kb)

## Abbreviations

GBM: Glioblastoma multiforme
iN: induced neurons
Inhibitor P: palomid 529
Inhibitor Y: Y27632
iPS: Induced pluripotent stem

## References

[1] Takahashi K, Tanabe K, Ohnuki M (2007). Induction of pluripotent stem cells from adult human fibroblasts by defined factors. Cell.

[2] Pang ZP, Yang N, Vierbuchen T (2011). Induction of human neuronal cells by defined transcription factors. Nature.

[3] Vierbuchen T, Ostermeier A, Pang ZP, Kokubu Y, Sudhof TC, Wernig M (2010). Direct conversion of fibroblasts to functional neurons by defined factors. Nature.

[4] Qiang L, Fujita R, Yamashita T (2011). Directed conversion of Alzheimer's disease patient skin fibroblasts into functional neurons. Cell.

[5] Caiazzo M, Dell'Anno MT, Dvoretskova E (2011). Direct generation of functional dopaminergic neurons from mouse and human fibroblasts. Nature.

[6] Pfisterer U, Kirkeby A, Torper O (2011). Direct conversion of human fibroblasts to dopaminergic neurons. Proc Natl Acad Sci U S A.

[7] Yoo AS, Sun AX, Li L (2011). MicroRNA-mediated conversion of human fibroblasts to neurons. Nature.

[8] Ambasudhan R, Talantova M, Coleman R (2011). Direct reprogramming of adult human fibroblasts to functional neurons under defined conditions. Cell Stem Cell.

[9] Son EY, Ichida JK, Wainger BJ (2011). Conversion of mouse and human fibroblasts into functional spinal motor neurons. Cell Stem Cell.

[10] Ring KL, Tong LM, Balestra ME (2012). Direct reprogramming of mouse and human fibroblasts into multipotent neural stem cells with a single factor. Cell Stem Cell.

[11] Kim J, Su SC, Wang H (2011). Functional integration of dopaminergic neurons directly converted from mouse fibroblasts. Cell Stem Cell.

[12] Izgi K, Canatan H, Iskender B (2017). Current status in cancer cell reprogramming and its clinical implications. J Cancer Res Clin Oncol.

[13] Powers S, Pollack RE (2016). Inducing stable reversion to achieve cancer control. Nat Rev Cancer.

[14] Lang JY, Shi Y, Chin YE (2013). Reprogramming cancer cells: back to the future. Oncogene.

[15] Warrell RP, Frankel SR, Miller WH (1991). Differentiation therapy of acute promyelocytic leukemia with tretinoin (all-trans-retinoic acid). N. Engl. J. Med.

[16] Hochedlinger K, Blelloch R, Brennan C (2004). Reprogramming of a melanoma genome by nuclear transplantation. Genes Dev.

[17] Ramos-Mejia V, Fraga MF, Menendez P (2012). iPSCs from cancer cells: challenges and opportunities. Trends Mol Med.

[18] Zhang X, Cruz FD, Terry M, Remotti F, Matushansky I. Terminal differentiation and loss of tumorigenicity of human cancers via pluripotency-based reprogramming. Oncogene. 2013;32:2249–60. 226010.1038/onc.2012.237PMC347078522777357

[19] Carette JE, Pruszak J, Varadarajan M (2010). Generation of iPSCs from cultured human malignant cells. Blood.

[20] Utikal J, Maherali N, Kulalert W, Hochedlinger K (2009). Sox2 is dispensable for the reprogramming of melanocytes and melanoma cells into induced pluripotent stem cells. J Cell Sci.

[21] Miyoshi N, Ishii H, Nagai K (2010). Defined factors induce reprogramming of gastrointestinal cancer cells. Proc.Natl.Acad.Sci.U.S.A..

[22] Chang G, Miao YL, Zhang Y (2010). Linking incomplete reprogramming to the improved pluripotency of murine embryonal carcinoma cell-derived pluripotent stem cells. PLoS.One.

[23] Choi SM, Liu H, Chaudhari P (2011). Reprogramming of EBV-immortalized B-lymphocyte cell lines into induced pluripotent stem cells. Blood.

[24] Hu K, Yu J, Suknuntha K (2011). Efficient generation of transgene-free induced pluripotent stem cells from normal and neoplastic bone marrow and cord blood mononuclear cells. Blood.

[25] Lin SL, Chang DC, Chang-Lin S (2008). Mir-302 reprograms human skin cancer cells into a pluripotent ES-cell-like state. RNA.

[26] Amson R, Pece S, Lespagnol A (2011). Reciprocal repression between P53 and TCTP. Nat Med.

[27] Amson R, Karp JE, Telerman A (2013). Lessons from tumor reversion for cancer treatment. Curr Opin Oncol.

[28] Papp B, Plath K (2011). Reprogramming to pluripotency: stepwise resetting of the epigenetic landscape. Cell Res.

[29] Ho R, Chronis C, Plath K (2011). Mechanistic insights into reprogramming to induced pluripotency. J Cell Physiol.

[30] Han SS, Williams LA, Eggan KC (2011). Constructing and deconstructing stem cell models of neurological disease. Neuron.

[31] Cherry AB, Daley GQ (2012). Reprogramming cellular identity for regenerative medicine. Cell.

[32] Robinton DA, Daley GQ (2012). The promise of induced pluripotent stem cells in research and therapy. Nature.

[33] Bleeker FE, Molenaar RJ, Leenstra S (2012). Recent advances in the molecular understanding of glioblastoma. J Neurooncol..

[34] Tamimi AF, Juweid M, Thakkar JP (2014). Epidemiology and Outcome of Glioblastoma. Epidemiologic and molecular prognostic review of glioblastoma. Cancer Epidemiol Biomarkers Prev..

[35] Young RM, Jamshidi A, Davis G, Sherman JH (2015). Current trends in the surgical management and treatment of adult glioblastoma. Ann Transl Med.

[36] Qin Y, Takahashi M, Sheets K (2017). Epithelial membrane protein-2 (EMP2) promotes angiogenesis in glioblastoma multiforme. J Neurooncol.

[37] Hingtgen S, Figueiredo JL, Farrar C (2013). Real-time multi-modality imaging of glioblastoma tumor resection and recurrence. J Neurooncol..

[38] Kauer TM, Figueiredo JL, Hingtgen S, Shah K (2011). Encapsulated therapeutic stem cells implanted in the tumor resection cavity induce cell death in gliomas. Nat Neurosci.

[39] Fomchenko EI, Holland EC (2006). Mouse models of brain tumors and their applications in preclinical trials. Clin Cancer Res.

[40] Jacobs VL, Valdes PA, Hickey WF, De Leo JA (2011). Current review of in vivo GBM rodent models: emphasis on the CNS-1 tumour model. ASN.Neuro.

[41] Collado M, Blasco MA, Serrano M (2007). Cellular senescence in cancer and aging. Cell.

[42] Yang Q (2008). Cellular senescence, telomere recombination and maintenance. Cytogenet Genome Res.

[43] Yang Q, Zhang R, Horikawa I (2007). Functional diversity of human protection of telomeres 1 isoforms in telomere protection and cellular senescence. Cancer Res.

[44] Beausejour CM, Krtolica A, Galimi F (2003). Reversal of human cellular senescence: roles of the p53 and p16 pathways. EMBO J.

[45] Campisi J (2005). Senescent cells, tumor suppression, and organismal aging: good citizens, bad neighbors. Cell.

[46] Utikal J, Polo JM, Stadtfeld M (2009). Immortalization eliminates a roadblock during cellular reprogramming into iPS cells. Nature.

[47] Li H, Collado M, Villasante A (2009). The Ink4/Arf locus is a barrier for iPS cell reprogramming. Nature.

[48] Sun CK, Zhou D, Zhang Z (2014). Senescence impairs direct conversion of human somatic cells to neurons. Nat Commun.

[49] Zhou D, Zhang Z, He LM (2014). Conversion of fibroblasts to neural cells by p53 depletion. Cell Rep.

[50] Wong CC, Wong CM, Au SL, Ng IO (2010). RhoGTPases and rho-effectors in hepatocellular carcinoma metastasis: ROCK N'Rho move it. Liver Int.

[51] Micuda S, Rosel D, Ryska A, Brabek J (2010). ROCK inhibitors as emerging therapeutic candidates for sarcomas. CurrCancer Drug Targets.

[52] Narumiya S, Tanji M, Ishizaki T (2009). Rho signaling, ROCK and mDia1, in transformation, metastasis and invasion. Cancer Metastasis Rev.

[53] Olson MF (2008). Applications for ROCK kinase inhibition. Curr Opin Cell Biol.

[54] Chen T, Shen L, Yu J (2011). Rapamycin and other longevity-promoting compounds enhance the generation of mouse induced pluripotent stem cells. Aging Cell.

[55] Menendez JA, Vellon L, Oliveras-Ferraros C, Cufi S, Vazquez-Martin A (2011). mTOR-regulated senescence and autophagy during reprogramming of somatic cells to pluripotency: a roadmap from energy metabolism to stem cell renewal and aging. Cell Cycle.

[56] Cornu M, Albert V, Hall MN. mTOR in aging, metabolism, and cancer. Curr Opin Genet Dev; 2013;23:53–62.10.1016/j.gde.2012.12.00523317514

[57] Kaeberlein M (2010). Lessons on longevity from budding yeast. Nature.

[58] Weichhart T (2012). Mammalian target of rapamycin: a signaling kinase for every aspect of cellular life. Methods Mol Biol.

[59] McCormick MA, Tsai SY, Kennedy BK (2011). TOR and ageing: a complex pathway for a complex process. Philos.Trans.R.Soc.Lond B Biol Sci.

[60] Harrison DE, Strong R, Sharp ZD (2009). Rapamycin fed late in life extends lifespan in genetically heterogeneous mice. Nature.

[61] Abbruzzese C, Catalogna G, Gallo E (2017). The small molecule SI113 synergizes with mitotic spindle poisons in arresting the growth of human glioblastoma multiforme. Oncotarget.

[62] Talarico C, Dattilo V, D'Antona L (2016). SI113, a SGK1 inhibitor, potentiates the effects of radiotherapy, modulates the response to oxidative stress and induces cytotoxic autophagy in human glioblastoma multiforme cells. Oncotarget.

[63] Agrawal R, Garg A, Benny MP, Sharma V, Sarkar C, Kulshreshtha R (2018). p53 and miR-210 regulated NeuroD2, a neuronal basic helix-loop-helix transcription factor, is downregulated in glioblastoma patients and functions as a tumor suppressor under hypoxic microenvironment. Int J Cancer.

[64] Park NI, Guilhamon P, Desai K (2017). ASCL1 reorganizes chromatin to direct neuronal fate and suppress Tumorigenicity of glioblastoma stem cells. Cell Stem Cell.

[65] Guichet PO, Guelfi S, Teigell M (2015). Notch1 stimulation induces a vascularization switch with pericyte-like cell differentiation of glioblastoma stem cells. Stem Cells.

[66] Hu J, Ho AL, Yuan L (2013). From the cover: neutralization of terminal differentiation in gliomagenesis. Proc Natl Acad Sci USA.

